The article "Comprehensive Landscape of Modules-Dysregulated Functions Reveals a Profound Role of ceRNAs in Coronary Heart Disease" was published in 2022. Journal: J Healthc Eng.

# Comprehensive Landscape of Modules-Dysregulated Functions Reveals a Profound Role of ceRNAs in Coronary Heart Disease

**DOI:** 10.1155/2022/4547413

**Published:** 2022-03-08

**Authors:** Chen Chen, Li Wang, Qiuju Feng, Qi Liu, Li Wang, Shuming Huang

**Affiliations:** ^1^Institute of Chinese Medicine, Heilongjiang University of Chinese Medicine, Harbin 150040, China; ^2^Harbin Traditional Chinese Medicine Hospital, Harbin 150076, China; ^3^College of Bioinformatics Science and Technology, Harbin Medical University, Harbin, China

## Abstract

Coronary heart disease (CHD) is one of the most common severe cardiovascular diseases. Competitive endogenous RNAs (ceRNA) play critical roles in complex diseases. However, our understanding of the dysregulated functions of ceRNAs in CHD remains limited. Here, we systematically analyzed the alterations of ceRNAs and identified the specific functions based on dysregulated modules from the ceRNA network. A total of 2457 significantly differential expressed genes and 212 differential expressed lncRNAs were identified. We got 76679 regulator relationship between different expression genes and miRNAs and 336 regulator relationship between differential expressed lncRNAs and miRNAs. We constructed the ceRNA network and selected five dysregulated modules. Furthermore, CHD specific functions based on dysregulated modules from the ceRNA network were identified, including histone acetylation, platelet degranulation, cAMP-dependent protein kinase complex, xenobiotic transport and so on. Our results will provide novel insight for a better understanding of the mechanism of ceRNAs and facilitate the identification of novel diagnostic and therapeutic biomarkers in CHD.

## 1. Introduction

Coronary heart disease (CHD) is one of the most common severe cardiovascular diseases [1]. CHD results from the buildup of plaques in the coronary arteries, and the ruptured plaques may induce thrombosis in coronary atherosclerosis [2, 3]. Despite remarkable success in the surgical and medical management of CHD, many interventions are palliative rather than curative, and some survivors still have significant residual hemodynamic and electrical conduction abnormalities and experience cardiovascular complications over the long term [4, 5]. The genetic susceptibility to CHD has aroused much attention. Studies have shown that more than 400 genes are associated with the incidence, pathogenesis, and progression of CHD [6, 7]. MicroRNAs (miRNAs) are a type of small noncoding RNA composed of 21–22 nucleotides [8, 9]. They exert their biological effects by silencing genes posttranscriptionally via binding to miRNA response elements (MREs) in the target mRNA [10, 11]. The report suggested that miR-451 is upregulated in CHD and is associated with the PI3K-Akt-mTOR pathway; the data indicated that miR-451 might be a novel biomarker for CHD [12]. Long noncoding RNAs (lncRNAs) defined as nonprotein-coding RNAs longer than 200 nucleotides [13]. Some studies verified that the abnormal expression of lncRNA in CHD [14–16]. Liu et al. reported that lncRNA-ANRIL is expressed low in the serum of patients with CHD, and it has high predictive value both for effective treatment and for poor prognosis of them. lncRNA-ANRIL is also an independent risk factor for patients poor prognosis [17, 18]. Competing endogenous RNAs (ceRNAs) are transcripts that can regulate each other at the posttranscription level by competing for shared miRNAs [19, 20]. Numerous studies have highlighted that lncRNAs can bind to miRNA sites as ceRNAs, thereby affecting and regulating the expression of mRNAs and target genes [21, 22]. One study observed that the direct binding between lncRNA-MEG3 and miR-26a was confirmed via dual-luciferase reporter assay, which indicated that lncRNA-MEG3 could sponge miR-26a as a ceRNA in CHD [23]. The other study provided evidence that lncRNA HIF1A-AS1 could act as ceRNA to adsorb miR-204 to suppress miR-204 expression and elevate SOCS2 expression in a mouse model, which was established by left coronary artery occlusion [24].

In the present study, based on the ceRNA hypothesis, we constructed a ceRNA network focused on CHD mechanisms and therapy opportunities by utilizing associated miRNA, lncRNA, and mRNA expression profiles. We constructed a ceRNA regulator network among lncRNA-miRNA-mRNA after acquiring the interaction relationship between miRNA and dysregulated genes and miRNA and dysregulated lncRNA. Drug treatment could influence the molecular network of disease mechanisms. Therefore, we constructed a ceRNA and drug-target interaction network based on the interaction network. Five functionally-related modules were identified from the ceRNA network. Dysregulated modules based on the ceRNA mechanism play an important role of controlling CHD-specific biological functions. Drugs involved in modules, which target multiple genes and are regulated by more than one miRNA and lncRNA, may become promising therapeutic targets. We presented a landscape of dysregulated ceRNAs acting as a valuable resource for the investigation of the relationship between ceRNA and CHD. Flowchart of the strategy to identify modules-based CHD specific functions is shown in Figure 1.

## 2. Materials and Methods

### 2.1. Expression Dataset of Coronary Heart Disease

Gene expression and lncRNA expression data were obtained from the exoRBase database (http://www exoRBase org) [25], which is a repository of lncRNA and mRNA derived from RNA-seq data analyses of human blood exosomes. All collected datasets were processed through a consistent bioinformatics pipeline. The expression profiles included a total of 38 samples, consisting of 6 disease samples and 32 normal samples. RNA-seq data standardized by TPM, expression profile transformed by log(*x*+1) for analysis.

### 2.2. Identification of Epigenetically Dysregulated lncRNAs and PCGs

Based on the expression data from the database, *t*-test and fold change [26] were applied to identify the different expression genes (DEGs) and different expression lncRNAs (DELs) among CHD and normal samples. The fold change value was calculated by the average expression of genes or lncRNAS in the disease sample divided by the average gene of genes or lncRNAS in the normal sample. After significance analysis and false discovery rate (FDR) adjusting, FDR <0.05 was considered as significant difference between DEGs and DELs.

### 2.3. Identifying ceRNA Regulatory Relationships

This report sets up ceRNA regulatory relationships in two steps. Firstly, we downloaded experimentally confirmed interaction relationship between miRNA and lncRNA, miRNA and target gene from starBase database (http://starbase sysu.edu cn/[27]), selected regulatory relationship between miRNA and DELs and miRNA and DEGs. These two types of relations performed hypergeometric to identify shared miRNA. The specific calculation formula is as follows:

(1) $$\begin{array}{c} P\text{ value}=1-\sum_{i-0}^{r-1}\frac{\left(t/i\right)\left(m-t/n-i\right)}{\left(m/n\right)}. \end{array}$$

Where *m* represents the total number of human miRNAs, *t* represents the number of miRNAs that interact with mRNA, *n* represents the number of miRNAs that interact with lncRNA, *r* represents the number of miRNAs shared mRNA and circRNA. By performing the hypergeometric test on the pairing relationship between mRNA and miRNA and the relationship between lncRNA and miRNA, we restricted FDR <0.05 and received a preliminary ceRNA relationship.

Secondly, studies have found that overexpression of lncRNA reduces the number of free miRNA molecules, which in turn leads to gene high expression which are targeted by miRNA. Coexpression is a common method for determining regulatory relationships. We calculated the Pearson's correlation, thus getting the corresponding correlation coefficient cor values of mRNA and lncRNA in normal samples and disease samples, respectively. Considering the statistical significance of the algorithm and the size of the network, we believed that the coefficient cor between mRNA and lncRNA in disease and normal samples is greater than 0.5 and the *p* value smaller than 0.05, which corresponds to the coexpression relationship. The mathematical formula is as follows:

(2) $$\begin{array}{c} \left|\text{cor}\left(\text{case}\right)-\text{cor}\left(\text{control}\right)\right|0.5. \end{array}$$

### 2.4. Identifying Dysregulated Modules of ceRNA Network

We constructed a ceRNA regulatory network based on the interaction data between miRNA and lncRNA, miRNA, and mRNA. The Cytoscape software was used for the construction of networks. Based on the ceRNA network, we identified modules using GraphWeb, a web server tool for identifying the network-based biomarkers that best represent the properties of the network [28]. The GraphWeb tools consisted of three component processes: network datasets (to input human protein-protein interaction pairs; ceRNA network in this present study); network algorithm (we used the betweenness centrality clustering method and the default values were set); and network settings (including default edge settings, node settings, and module settings with less than 3 nodes and insignificant modules hidden). It has recently been reported that the emerging ceRNA networks are involved in drug resistance of disease [29]. In order to explore the interaction between drugs and ceRNA. Furthermore, we downloaded all drug-targeted data from the DrugBank database (https://www drugbank ca/) [30], matched the genes in the ceRNA network and modules with the drug-target genes, and added the drugs that target the genes in the ceRNA network and modules, obtaining a ceRNA network and modules that include drug information.

### 2.5. CHD Specific Functions Annotation Analysis of Dysregulated Modules

Biological function annotation analysis of genes in the network and each module at the Gene Ontology GO (http://geneontology.org/33290552) levels was performed by using the *R* package clusterProfiler. clusterProfiler provides a universal interface for gene functional annotation from a variety of sources. clusterProfiler from website bioconductor, it can directly find the enriched gene entrez ID number based on cuffdiff and find the difference [31].

## 3. Results

### 3.1. Identifying Dysregulated lncRNAs and PCGs in CHD

We obtained 16225 genes and 1735 lncRNA expression profiles from the exoRBase database. Firstly, we used *T*-test and fold change to identify 2457 DEGs and 212 DELs compared to normal samples. The ratio of DEGs to all genes is 15% (Figure 2(a)), and the ratio of DELs to all lncRNAs is 12% (Figure 2(b)). For DEGs and DELs, we found that there are differences in expression levels between CHD and normal samples. Some genes are upregulated in normal samples and downregulated in CHD samples, but other genes are opposed (Figure 2(c) and Figure 2(d)). Significantly downregulated DEGs TRIM69 has been affirmed that is associated with heart failure (Figure 2(e)). They used robust rank aggregation to derive an integrative transomic score for each annotated gene associated with a heart failure trait, TRIM69 for incident HF with reduced ejection fraction [32]. We also identified significantly upregulated and downregulated DELs (Figure 2(f)).

Yan et al. suggested that lncRNA necrosis-related factor (NRF) was shown to be increased in acute myocardial infarction (AMI) patients with heart failure compared with AMI patients without heart failure and had predictive value for the diagnosis of heart failure [33]. The report also suggested that lncRNA SNHG14 (small nucleolar RNA host gene 14) was validated to sponge both miR-322-5p and miR-384-5p to elevate PCDH17 levels in vivo and in vitro cardiac hypertrophy models. The subsequent rescue assays revealed that miR-322-5p and miR-384-5p restored SNHG14 depletion-mediated suppression on hypertrophy in Ang–II–induced cardiomyocytes [34].

### 3.2. Characterizing ceRNA Relationship and Constructing Network in CHD

We obtained 10212 pairs interactions between lncRNA and miRNA, 423975 pairs interactions between genes and miRNA from the starBase database, and selected 336 pairs interactions between DELs and miRNA and 76679 pairs interaction between DEGs and miRNA. We identified 6334 lncRNA and gene pairs that shared miRNA after applied hypergeometric. Then, we used coexpression identified expression-regulated lncRNA and gene pairs. We finally got an lncRNA-miRNA-mRNA regulator relationship as a candidate ceRNA and constructed a ceRNA network based on the regulator relationship among lncRNA, miRNA, and mRNA. Furthermore, we added drug information into the network based on the DrugBank (Figure 3).

By integrating lncRNAs-miRNA interactions, mRNAs-miRNA interactions, and drug-target relationships, the ceRNA network was constructed. The network included 1407 edges and 290 nodes, respectively, 13 lncRNAs, 139 miRNAs, 90 mRNAs, and 48 drugs. Some genes are targeted by multiple drugs, such as PDE4D. lncRNA linc00867, with a high degree, may play an important role in the ceRNA network. We identified that miRNA hsa-miR-224-5p targeted gene MAPKAPK2, lncRNA LINC00665 regulated miRNA hsa-miR-224-5p in CHD patients, and hsa-miR-224-5p was shared between LINC00665 and MAPKAPK2. At the same time, the nodes of LINC00665 and MAPKAPK2 have a relatively high degree in networks. Therefore, ceRNA regulator relationship among LINC00665, hsa-miR-224-5p, and MAPKAPK2 was identified. From the DrugBank database, we got the small molecule drug staurosporine, that is, a potent protein kinase C inhibitor which enhances cAMP-mediated responses in human neuroblastoma cells [35]. This present study suggested that staurosporine influenced ceRNA relationship LINC00665-hsa-miR-224-5p-MAPKAPK2 through targeted gene MAPKAPK2.

### 3.3. Identifying Dysregulated Modules Based on ceRNA Network in CHD

We identified five modules based on the ceRNA network by GraphWeb (Figure 4). In each module, we have identified many key nodes. Such as in module2 (Figure 4(b)), gene TMX3 downregulated in CHD samples compared to normal samples, FC value equal to 0.41, lncRNA NUTM2A-AS1 FC value equal to 0.47. Downregulated lncRNA LINC00665 FC value equal to 0.40, meanwhile gene PRKG1 FC value is 0.49 in module4 (Figure 4(d)). In module5, linRNA TAPT1-AS1 FC value is 0.25 and gene SOCS5 FC value is 0.41 (Figure 4(e)). Li et al. used whole-exome sequencing (WES) to explore pathogenic variants present in a Zhuang family with coronary artery disease, they discovered two pathogenic mutations, PPP2R3A and TMX3 in four members of the CHD group and two members of the high-risk group [36]. The elements in each module have a close regulatory relationship. In module1, we found the regulated relationship among hub nodes OIP5-AS1-has-mir-153-3p-CREBBP, and in module2 we identified ceRNA relationship NUTM2A-AS1-hsa-mir-107-PDE4D, iloprost is a small molecule drug that was used to treat pulmonary arterial hypertension (PAH) through regulated target gene PDE4D [37].

Our study suggested that the drug iloprost impacted ceRNA among NUTM2A-AS1, hsa-mir-107 and PDE4D. LINC00667 is hub node in ceRNA network, we found some ceRNA relationships including LINC00667 in module3 (Figure 4(c)). In our work, to explored the relationship between ceRNA network and drug, we identified functionally modules (ceRNA-drug) to explored the relationship between ceRNA network and drug. For instance, module4 contains various ceRNA interactions, involving the hub gene MAPKAPK2. Many genes, such as CMPK1, PDE4D, and MAPKAPK2, are targeted by multidrugs. Moreover, other studies have reported that the PDE4D gene interacts with serum triglyceride, and the haplotypic association found in the present population is indicative of the population-specific risk associated with CHD [38]. Thus, we considered using drugs that targeted the gene PED2D for the treatment of CHD patients.

### 3.4. Dysregulated Modules of the ceRNAs Network Contributing to CHD Specific Functions

We performed function enrichment analysis based on the whole ceRNA network and five dysregulated modules in CHD (Figure 5). Myeloid cell differentiation and histone acetyltransferase have been discerned in the ceRNA network (Figure 5(a)), meanwhile other reports also suggested ceRNA regulated myeloid cell differentiation. Cheng et al. reported that ceRNA regulated relationship influenced histone acetyltransferase binding function [38], confirming the reliability of dysregulated modules in our results. We obtained 10 biological functions from module 1, such as histone modification and acetylation, other researches have reported that aberrant histone modifications, including acetylation and trimethylation, were found both in global histone and specific MCP-1 gene locos in monocytes from patients with CHD (Figure 5(b)). Aberrant epigenetic modification enzymes expression may be the regulatory mechanism responsible for aberrant histone modifications [39, 40]. In module2, platelet degranulation pathway was identified, at the same time, other reports suggested anticoagulated peripheral venous blood from 19 patients with stable CHD and 19 normal control subjects was incubated with or without various platelet agonists and analyzed by whole blood flow cytometry, and it turns out that circulating degranulated platelets were increased in patients with CHD compared with control subjects (Figure 5(c)) [41]. Some studies on account of high-throughput gene expression data have also shown that platelet degranulation is associated with CHD [42].

More interestingly, we also identified several KEGG pathways related to CHD, vascular smooth muscle contraction identified in network (Figure 6(a)), ovarian steroidogenesis identified in module2 (Figure 6(b)), and prolactin signaling pathway identified in module5 (Figure 6(c)). Some genes are linked with multiple genes in the ceRNA network. These hub genes participated in many ceRNA regulator relationships. For instance, the hub gene CREBBP from module1 plays an important role in CHD, and studies have indicated that CITED2, which encodes a CREBBP/EP300 interacting transcriptional modulator of HIF1A and TFAP2, has a causative impact in the development of CHD in humans [43]. In module2, hub gene GNAS interacted with many miRNAs and lnRNAs, GNAS-EDN3 gene loci is associated with hypertension, left ventricular wall thickness, stroke and coronary artery disease based on 29 genome-wide significant variants [44].

Therefore, hub genes which are involved in lots of ceRNA relationships may affect many CHD-related specific biological functions, in turn influencing the progression of coronary heart disease. Our work conducted ceRAN network-related drugs in CHD, and identified five functionally-related modules from the ceRNA network. Drugs involved in functionally-related modules, which target multiple genes and are regulated by more than one miRNA and lncRNA, may become promising therapeutic targets.

## 4. Discussion

The majority of patients with CHD are diagnosed at advanced stages and have poor overall survival. Thanks to high-throughput sequencing technology and the rapid development of bioinformatics, we are able to discover the various aberrant expressions of RNAs in disease samples. Unlike classic molecular or cellular biology studies that focus on a specific molecular interaction, the ceRNA network is constructed to provide a more comprehensive view of the RNA regulatory mechanism during CHD. Current databases have the apparent advantage that they contain multifarious high-throughput data types. This enables researchers to discover changes between different kinds of RNA and to uncover the regulatory mechanisms between the ceRNAs. Therefore, our study used expression and regulation data from the exoRBase and starBase databases to identify ceRNA relationship pairs related to coronary heart disease, and applied drug-target information from DrugBank to build a ceRNA drug network. Mined modules from the network and identified functional pathways related to the network and modules.

## 5. Conclusions

In conclusion, the present study constructed a novel ceRNA regulator network including some drug information. The network may be associated in the progression of CHD. We also mined CHD specific functions and pathways from dysregulated five modules of the ceRNAs network which may be associated in the progression of CHD. However, the sample size of CHD is not large, and the data types are not sufficient, such as clinical data and prognostic information. In the future, if more types of data are available, it will be beneficial to the study of the mechanism of coronary heart disease.

## Figures and Tables

**Figure 1:** Flowchart of the strategy to identify modules-based CHD specific functions.

**Figure 2:** Differential expression of normal samples and disease samples in CHD. (a, b) The pie chart represents the radio of differentially expressed mRNAs and lncRNAs. (c, d) The heatmap chart of expression of DEGs and DELs in CHD and normal samples; rows represent DEGs or DELs and columns represent samples. (e, f) The volcano represents the significance level of DGEs and DELs.

**Figure 3:** Overview of the ceRNA network in CHD. Blue nodes represent miRNA, yellow nodes represent lncRNA, orange nodes represent mRNA, and green nodes represent drugs.

**Figure 4:** Dysregulated modules from the ceRNA network in CHD. (a) Module1, (b) module2, (c) module3, (d) module4, (e) and module5. Blue nodes represent miRNA, yellow nodes represent lncRNA, orange nodes represent mRNA, and green nodes represent drugs.

**Figure 5:** CHD specific functions for dysregulated modules of ceRNAs network. (a) The ceRNA network annotation in GO categories. (b) Module1, (c) module2, (d) module3, (e) module4, and (f) module5 annotation in different biological function. The horizontal axis represents the score of ceRNA. The vertical axis represents different GO categories and biological functions. The bubble size indicates the number of genes in each category and biological function, and different colors correspond to different log (FDR) values.

**Figure 6:** CHD related pathways for dysregulated modules of ceRNAs network. (a) The network, (b) module2, and (c) module5 enrichment function. The horizontal axis represents the score of ceRNA. The vertical axis represents different KEGG function pathways. The bubble size indicates the number of genes in each category and pathway, and different colors correspond to different log (FDR) values.

## Data Availability

Gene expression and lncRNA expression data were obtained from the exoRBase database (http://www exoRBase org).
